The article "Thoracic myelopathy caused by ossification of ligamentum flavum of which fluorosis as an etiology factor" was retracted in 2007. Reasons: duplicate publication; a breach of policy by an author.

# Thoracic myelopathy caused by ossification of ligamentum flavum of which fluorosis as an etiology factor

**DOI:** 10.1186/1749-799X-1-10

**Published:** 2006-11-02

**Authors:** Wenbao Wang, Linghua Kong, Heyuan Zhao, Ronghua Dong, Jing Zhou, Yun Lu

**Affiliations:** 1 Spine surgery department, Tianjin hospital, No. 406 Jiefangnan Road, Hexi District, Tianjin City, 300211, People's Republic of China; 2 106 Fort Washington Avenue, Room 3H, New York City, NY, 10032, USA; 3 Hand surgery department, Tianjin hospital, No. 406 Jiefangnan Road, Hexi District, Tianjin City, 300211, People's Republic of China

## Abstract

**Purpose:**

To evaluate the clinical feature, operative method and prognosis of thoracic ossification of ligamentum flavum caused by skeletal fluorosis.

**Methods:**

All the patients with thoracic OLF, who underwent surgical management in the authors' hospital from 1993–2003, were retrospectively studied. The diagnosis of skeletal fluorosis was made by the epidemic history, clinical symptoms, radiographic findings, and urinalysis. En bloc laminectomy decompression of the involved thoracic levels was performed in all cases. Cervical open door decompression or lumbar laminectomy decompression was performed if relevant stenosis existed. The neurological statuses were evaluated with the Japanese Orthopaedic Association (JOA) scoring system preoperatively and at the end point of follow up. Also, the recovery rate was calculated.

**Results:**

23 cases have been enrolled in this study. Imaging study findings showed all the cases have ossification of ligamentum flavum together with ossification of many other ligaments and interosseous membranes, i.e. interosseous membranes of the forearm in 18 of 23 (78.3%), of the leg in 14 of 23 (60.1%) and of the ribs in 11 of 23 (47.8%). Urinalysis showed markedly increased urinary fluoride in 14 of 23 patients (60.9%). All the patients were followed up from 12 months to 9 years and 3 months, with an average of 4 years and 5 months. The JOA score increased significantly at the end of follow up (P = 0.0001). The recovery rate was 51.83 ± 32.36%. Multiple regression analysis revealed that the preoperative JOA score was an important predictor of surgical outcome (p = 0.0022, r = 0.60628). ANOVA analysis showed that patients with acute onset or too long duration had worse surgical result (P = 0.0003).

**Conclusion:**

Fluorosis can cause ossification of thoracic ligamentum flavum, as well as other ligaments. En bloc laminectomy decompression was an effective method. Preoperative JOA score was the most important predictor of surgical outcome. Patients with acute onset or too long duration had worse surgical outcome.

The article "Thoracic myelopathy caused by ossification of ligamentum flavum of which fluorosis as an etiology factor" was retracted in 2007. Reasons: duplicate publication; a breach of policy by an author.

## Background

Fluoride is an important element for bone mineralization. It causes an increase in bone mass by stimulation of the osteogenetic process [1]. However, over intake of fluoride may cause fluoride intoxication, so-called fluorosis [2-10]. Its typical clinical features include dental fluorosis, diffuse densification of bone, calcifications of bony insertions of many ligaments, discs, and interosseous membranes, *i.e*. interosseous of the ribs, forearm, and leg, posterior longitudinal ligament, transverse atlantal ligament, ligamentum flavum, and membrana obturatoria [8-10]. Thoracic spinal stenosis caused by ossification of ligamentum flavum (OLF) is a rare disease [11-20]. However, thoracic OLF caused by skeletal fluorosis is rather rare. Only 6 cases have been reported in the English literature [3,13]. The authors' purpose is to evaluate the clinical feature, operative method, and prognosis of thoracic OLF caused by skeletal fluorosis.

## Materials and methods

All the patients with thoracic OLF, who underwent surgical management in the authors' hospital from 1993–2003, were retrospectively studied. The cases accorded with the following criteria were included. Diagnostic criteria for fluorosis: epidemic history including a long history living in a high fluorosis area; dental fluorosis; typical X-ray findings including diffuse densification of bone, calcifications of bony insertions of many ligaments, discs, and interosseous membranes, *i.e*. interosseous of ribs, forearm, and leg; urinalysis of fluoride may increase. Diagnostic criteria for thoracic ossification of ligamentum flavum: typical clinical symptoms and findings which included numbness in the lower limbs and below the relative segment of trunk, motor weakness in the lower extremities and difficulty in walking; physical examination showed increased lower limbs muscle tension, increased in deep tendon reflexes and appearance of pathological reflex, i.e. Babinski sign. X ray, CT scan, and MRI were used to confirm the diagnosis.

For each the patient, A-P view and lateral view X-ray of the thoracic spine were taken. Then thoracic MRI was taken to ensure the diagnosis and identify the involved segments. CT scan was performed for the involved segments. A-P view, lateral view X-ray of forearms and legs and A-P view of the chest were also taken.

Indication of surgery: symptoms and signs of thoracic myelopathy; CT scan and MRI demonstrated significant thoracic canal stenosis; the symptoms and signs correlation with the imaging findings.

En bloc decompression was performed on each patient. In one patient combined with cervical ossification of posterior longitudinal ligament, cervical open door decompression was performed additionally. In one patient combined with lumbar stenosis, lumbar laminectomy decompression was performed additionally.

The article "Thoracic myelopathy caused by ossification of ligamentum flavum of which fluorosis as an etiology factor" was retracted in 2007. Reasons: duplicate publication; a breach of policy by an author.

Preoperative radiographic localization with a Kirschner wire was used to confirm the operative level on the morning of operation day. After induction of general anesthesia, the patient was placed prone with an indwelling bladder catheter. The abdomen was decompressed to avoid excessive epidural bleeding. According to the X-ray localization result, a midline incision was made at the appropriate level and extended to the fascia. Subperiosteal dissection of the paraspinal muscles was performed using electrocautery cutting. The spinous processes were shortened using rongeurs (not totally removed). The laminectomy was performed with high-speed drill. The width of the laminectomy was approximately one third the size of the inside of the facet. After the laminae were totally floated, it was taken off en bloc by holding the residues spinous processes (Fig 4).

The ossified ligamentum flavum often adhered to the dura mater. So, much care should be paid to avoid rupture of the dura mater. Occasionally, the dura mater also ossified. In those cases, we did not take away the ossified dura mater totally, just floated it. When coexistent lesions were present at noncontinuous thoracic levels, clinical symptoms and neuro-imaging findings were examined. The level considered to be the likely cause of clinical symptoms was then surgically treated. When coexistent lesions were present at the cervical or lumbar region, the depression of the relevant region was performed.

The neurological statuses were evaluated with the JOA scoring system of myelopathy preoperatively and at the end point of follow up (table 2). The recovery rate, described by Hirabayashi et al [21], indicating the degree of recovery of normal function postoperatively, was calculated as follows: (postoperative JOA score – preoperative JOA score)/(11- preoperative JOA score) ×100.

**Table 1:** Summary of clinical features observed in 23 patients with OLF

Symptoms	number of cases
numbness and sensory deficit	22
lower-limb weakness and gait disturbance	21
Low-back pain	8
"squeezing tight band" around chest or abdomen	6
neurological claudication	4
leg pain	12
fecal & urinary incontinence	18
knee and ankle hyperreflexia	18
positive patellar and ankle clonus	14
positive Babinski sign	15

**Table 2:** summary of the JOA scoring system for the assessment of myelopathy

neurological status	score
lower-limb motor dysfunction	
unable to walk	0
Able to walk on flat floor with walking aid	1
Able to walk up/downstairs w/handrail	2
Lack of stability & smooth reciprocation of gait	3
no dysfunction	4
lower-limb sensory deficit	
severe sensory loss or pain	0
Mild sensory deficit	1
no deficit	2
trunk sensory deficit	
severe sensory loss or pain	0
Mild sensory deficit	1
no deficit	2
sphincter dysfunction	
unable to void	0
marked difficulty in micturition	1
minor difficulty in micturition	2
no dysfunction	3

Total score for a healthy patient is 11.

The article "Thoracic myelopathy caused by ossification of ligamentum flavum of which fluorosis as an etiology factor" was retracted in 2007. Reasons: duplicate publication; a breach of policy by an author.

X-ray and CT scan were performed 3 days after the operation to conform the decompression levels and decompression area. X-ray was performed at the end of the follow up to identify whether there was spinal instability.

### Statistical analysis

Paired t test was used to analyze the differences between the results before operation and at end of follow up. Multiple linear regression was conducted to determine the quantitative variables best correlating to surgical outcome. ANOVA was used to analyse differences among the three groups according to the duration of preoperative symptom. When the results of ANOVA indicated < 0.05, further statistical analysis was followed to determine whether there was any significance difference between any two groups. The statistical results were analyzed using the Statistical Analysis System (SAS). Significance was accepted for P-values of < 0.05 in all of the above analyses.

## Results

### Clinical presentation

74 cases of thoracic OLF were surgically treated at the authors' institution between 1993 and 2003, 23 of which (16 male and 7 female) were caused by fluorosis. The 23 patients ranged in age from 42 to 72 years (mean 54.8 years). 6 cases had acute onset of clinical symptom, 4 of which had a traumatic history, 2 without markedly traumatic history. The other 17 cases did not have a traumatic history and presented with progressive symptoms. Numbness in the lower limbs and below the relative segmental was the most common initial symptom in 17 of the 23 patients (73.9%). Motor weakness in the lower extremities and difficulty in walking as initial symptoms were found in 6 patients. The details of the clinical findings are shown in table 1 and table 3. The mean duration of symptoms between initial onset and operation was 37 months (range 1 day–11 years). All of the 23 patients had a long term, high fluoride area living history. Fluoride over intake was from water in 21 cases (91.3%) or from coal smoke in 2 cases (8.7%). 22 of 23 patients (95.7%) had different levels of dental fluorosis. Urinalysis showed markedly increased urinary fluoride in 14 of 23 patients (60.9%).

**Table 3:** Data on Patients With Ossification of Ligamentum Fluvam

case no.	sex & age	DPS & group	JOA score										levels & segment number of OLF	levels & number of decompression	recovery rate %
						
			pre-operation					follow up							
			LEM	TS	LES	SD	Total	LEM	TS	LES	SD	total			
1	M, 42	15m(2)	2	2	0	1	5	4	2	1	2	9	T12–L1 (1)	T12–L1 (2)	67
2	M,62	3d(1)	3	2	1	3	9	4	2	1	3	10	T12–L1 (1)	T12–L1 (2)	50
3	F, 46	32m(2)	3	1	1	2	7	4	2	1	3	10	T12–L1 (1)	T12–L1 (2)	75
4	M,54	12m(2)	4	1	1	3	9	4	2	2	3	11	C7–T1(1)	C7–T1(2)	100
5	F,64	4y(2)	2	1	1	2	6	4	2	1	3	10	T1–4(3)	T1–4(4)	80
6	M,51	5y(3)	1	1	0	2	4	3	2	1	3	9	T3–5(2)	T3–5(3)	71
7	M,42	2d(1)	1	1	0	1	3	2	2	1	2	7	T7–12(5)	T7–12(6)	50
8	M,65	7y(3)	1	1	1	1	4	3	1	1	1	6	T8–L1(5)	T8–T12(5)	29
9	M,55	11y(3)	2	1	1	3	7	2	2	1	3	8	T7–L1(5)	T8–L1(6)	25
10	F,56	15m(2)	2	1	1	2	6	3	2	1	2	8	T9–L1(4)	T10–L1(4)	40
11	M,59	1d(1)	2	1	0	1	4	2	1	0	1	4	T9–L1(4)	T9–L1(5)	0
12	M,45	6m(2)	4	2	1	3	10	4	2	2	3	11	T10–L1(3)	T10–L1(4)	100
13	F,50	5y(3)	2	2	1	1	6	3	2	1	2	8	T10–L1(3)	T10–L1(4)	40
14*	M,62	1d(1)	0	0	0	0	0	0	0	0	0	0	T10–L1(3)	T10–L1(4)	0
15	M,50	18m(2)	2	2	1	3	8	4	2	2	3	11	T10–L1(3)	T10–L1(4)	100
16*	F,48	5y(3)	2	1	1	2	6	2	1	1	2	6	T10–L1(3)	T10–L1(4)	0
17	M,54	1d(1)	0	1	0	1	2	0	1	0	2	3	T3–7		11
													T10–L1(4+3)	T10–L1(4)	
18	M,59	8y(3)	2	1	1	2	6	4	2	1	2	9	T1–T5	T1–T5(5)	60
													T9–L1(4+4)		
19	M,58	7y(3)	1	0	0	1	2	2	1	1	2	6	T1–6		44
													T9–L1(5+4)	T9–L1(5)	
20	M,56	6d(1)	2	1	1	1	5	3	1	1	2	7	C7–T9(9)	C7–T4(5)	33
21	F,52	7m(2)	2	1	1	2	6	4	2	2	3	11	T8–12(4)	T8–12(5)	100
22	F,72	7y(3)	2	2	1	1	6	4	2	1	2	9	T9–11	T9–11	60
													L3–S1(2+3)	L3–S1(3+4)	
23	M,58	4y(2)	1	1	0	2	4	3	2	1	2	8	C3–6	C3–6	57
													T10–L1(4+3)	T10–L1(4+4)	

DPS: duration of preoperative symptom. LEM: lower extremity motor; TS: trunk sensory; LES: lower extremity sensory; SD: sphincter dysfunction Paired t test showed that there is significant difference between the JOA score of pre-operation and followed up (P = 0.0001). The mean recover rate is 51.83%. ANOVA analysis of the three groups according to the DPS showed p = 0.0003. Further t test showed that there was significant different between group one and group tow (P = 0.0004). There was significant different between group two and group three (P = 0.003). However, there was no significant different between group one and group three (P = 0.197).

The article "Thoracic myelopathy caused by ossification of ligamentum flavum of which fluorosis as an etiology factor" was retracted in 2007. Reasons: duplicate publication; a breach of policy by an author.

### Imaging study result

The mean number of involved segments is 4.17, with a range from 1 to 9 (Fig 1). The ossified ligamentum flavum displayed obscuration the margin of the lamina on the A-P view X-ray in 8 patients (34.8%). On the lateral view X-ray, 12 of 23 patients (52.2%) showed high density projection into the spinal canal at the level of compression. All the ossified ligamentum flavum displayed the density of cortical bone on CT scans and sometimes had a thin gap between the laminae (Fig. 3c). All the ossified ligamentum flavum demonstrated triangular protrusion with a low-signal intensity resembling cortical bone on MR images (Fig 3a, 3b).

**Figure 1:** A diagram of the OLF distribution of 23 patients.

**Figure 2:** Anteroposterior view radiograph of both forearms showed significant calcifications of interosseous membranes of forearm.

**Figure 3:** a, b. T1 and T2 weight MRI of thoracic spine showed continuous multi-level ossification of ligamentum flavum between T7–12. c. CT scan showed ossified ligamentum flavum, note that there was a thin gap between the ossified ligament and the lamina.

**Figure 4:** The en bloc removed lamina, note the nodular ossified ligamentum flavum.

X-ray of forearms, legs, and chest showed ossification of interosseous membranes of the forearm in 18 of 23 patients (78.3%) (Fig 2), of the leg in 14 of 23 patients (60.1%), and of the ribs in 11 of 23 patients (47.8%).

### Operation and the prognosis

The operation time ranged from 2.5 hours to 4.3 hours, with a mean of 3.2 hours. The mean decompressed segments number is 4.35 (ranged from 2 to 8, table 3). Blood loss ranged from 400 ml to 2800 ml, with a mean of 850 ml. Dura mater rupture occurred in 4 patients. Deep infection occurred in one patient. No postoperative neurological deterioration occurred. All the patients were followed up from 12 months to 9 years and 3 months, with an average of 4 years and 5 months. Paired t test showed that the JOA score increased significantly at the end of follow up (P = 0.0001, table 3). The recovery rate was 51.83 ± 32.36%. Multiple regression analysis revealed that the preoperative JOA score was an important predictor of surgical outcome (p = 0.0022, r = 0.60628, table 4). However, the sex, age, preoperative symptom duration, and levels of OLF did not significantly influence the surgical outcome. ANOVA analysis showed that patients with acute onset (group 1) or too long duration (group 3) had worse surgical result (P = 0.0003) (table 3). Further t test showed that there was significant different between group 1 and group 2 (P = 0.0004). There was significant different between group 2 and group 3 (P = 0.003). However, there was no significant different between group 1 and group 3 (P = 0.197) (table 3). No postoperative instability occurred.

**Table 4:** results of a multiple linear regression analysis of selected variables to predict surgical outcome

	recover rate at final follow up	
	
Variable	coefficient	p value
Age	-0.24755	0.2548
duration of preoperative symptom	-0.10367	0.6378
Preoperative JOA score	0.60628	0.0022
levels of OLF	-0.31515	0.1430

## Discussion

### Etiology

The thoracic OLF was first reported by Polgar [17] in 1920 with lateral radiographs. From then on, several clinical series and many case reports have been reported. However, the etiology of OLF was unclear. As most of the reported OLF's were located between T9 and T12, Barnett et al. [11] suggested that the hyper mobility of the lower thoracic spine might promote degeneration and canal stenosis. Liao's study [22] showed a high prevalence of coexisting anterior osteophytes and herniated intervertebral disc at the symptomatic OLF segments. So they concluded that OLF might be a degenerative response to the micro injury of the ligamentum flavum. The hypothesis was histologically supported by Okada and colleagues [15] who found that OLF formed in the hypertrophic ligamentum flavum with fibrocartilage proliferation, and this was thought to be a phenomenon of mechanical injury. Therefore, it was thought that the development of OLF might be secondary to the specific fiber reconstruction of the ligamentum flavum in response to mechanical stress. However, Muthukumar [13] reported two cases of OLF caused by fluorosis, recently. Wang et al. [8-10] reported fluorosis could cause ossification of a lot of ligaments. All these reports showed fluorosis might play a role in OLF.

The article "Thoracic myelopathy caused by ossification of ligamentum flavum of which fluorosis as an etiology factor" was retracted in 2007. Reasons: duplicate publication; a breach of policy by an author.

Fluoride is one of the necessary minor elements for humans, and the daily requirement is 0.05–0.07 mg/kg body weight/day [2,5]. The benefits of water fluoridation in controlling dental caries were well documented. Fluoride was first used in water for caries control in 1945 and 1946 in the United States [1] and Canada [4], respectively. However, over intake of fluoride will cause fluorosis [2-10]. Fluorosis caused by fluoride intoxication was first reported by Feil in 1930, and skeletal fluorosis was reported by Short in 1937 [7]. Normally, there are two sources of fluoride over intake, water and coal smoke. In the high fluoride area, the density of fluoride in the water is more than 5–8 mg/L, and the people drink the water directly from the well without any management. This will cause dental fluorosis, skeletal fluorosis, or even systemic fluorosis.

It was reported that neurological complications occurred in approximately 10% of patients with skeletal fluorosis, usually in the later stages of the disease [7]. To date, the myeloradiculopathy caused by skeletal fluorosis was thought to be a result of compression of the spinal cord by osteophytes and vertebral osteosclerosis [7,23]. However, myelopathy caused by OLF in patients with skeletal fluorosis has been recognized recently [3,13]. So, we think fluorosis should be entertained as an etiology factor of OLF, especially in patients from endemic areas.

The pathogenesis of ossification of the ligaments in this condition remains speculative. High expression of transforming growth factor beta-1 (TGF-β1) by fibroblasts was found in the ossified matrix within ossified ligaments and in chondrocytes within cartilaginous areas adjacent to the ossified ligaments [24]. TGF-β1 could have played a role in chondroid metaplasia and ectopic ossification in OLF. Recent experimental evidence points to the involvement of proto-oncogenes c-fos and c-jun in skeletal fluorosis. Zhang et al. [25] have demonstrated that exposure to excessive fluoride could stimulate the activation and proliferation of osteoblast-like cells with enhanced expression of messenger ribonucleic acid and proteins of c-fos and c-jun.

The article "Thoracic myelopathy caused by ossification of ligamentum flavum of which fluorosis as an etiology factor" was retracted in 2007. Reasons: duplicate publication; a breach of policy by an author.

### Clinical feature of thoracic ossification of ligamentum flavum

Thoracic OLF is rare and usually asymptomatic. The disease usually has an insidious onset and very slow progression. Analysis of previously published epidemiological data reveals that thoracic OLF most commonly involves the vertebrae between T-9 and T-12(as in our serious in figure 1), where greater mobility and vulnerability (due to spinal motion) may result in frequent mechanical injury.

In our series, numbness in the lower limbs and below the relative segmental was the most common initial symptom in 17 of the 23 patients (73.9%). Motor weakness in the lower extremities and difficulty in walking as initial symptoms were found in 6 patients (26.1%). This finding is in agreement with the observations reported in previous studies [11-20]. When an extradural compressive lesion develops at the thoracic level, pressure to the spinothalamic tract, fasciculus gracilis and fasciculus cuneatus causes the numbness and lost of proprioceptive sensation in the lower limbs and below the relative segment. Upper neuron injury might occur and be caused by pressure to the cerebrospinal tract. This results in increasing muscle tension of the lower extremity, increasing in both patellar and Achilles reflexes. However, if at a lower thoracic level, the lesions exist at neighboring sites of the conus medullaris, the patellar or Achilles reflex will occasionally dissociate, or both decrease. Compressive coexistent lesions, such as cervical or/and lumbar stenosis, also influence the clinical features, as showed in the literature [26] and in our series. Although the neurological findings in our series are similar with other authors' findings, OLF caused by fluorosis has their own features. Firstly, all the patients had the character features of fluorosis. Secondly, the segment number of involved LF is more than others (figure 1).

### Surgical procedures

Non operative method is not effective for symptomatic patients. So, early diagnosis and operation interference were recommended for the symptomatic patients. As the thoracic OLF compressed the spinal cord posteriorly, several posterior decompression methods were developed. These operative techniques include open-door laminectomy, en bloc laminectomy, fenestration, total decompression et al. [14,15,18-20]. In our cases, all the patients performed en bloc decompression. The segments are shown in table 3. The blood loss was much more when compared with our non-fluorosis cases (non published data). This was partly because the fluorosis made the soft tissue easily prone to bleeding and partly because the decompression segments are more than others. The results shown in table 3 stated that the decompression was effective.

The article "Thoracic myelopathy caused by ossification of ligamentum flavum of which fluorosis as an etiology factor" was retracted in 2007. Reasons: duplicate publication; a breach of policy by an author.

In 4 cases of our patients, ossification of dura mater occurred. Some authors also reported ossification of the dura mater together with the ossification of thoracic ligamentum flavum [14]. In those cases, severe adhesion between ossified ligamentum flavum and dura mater might occur. Much attention must be paid to avoid rupture of the dura mater. However, some times we did not remove the ossified ligament totally. We just floated it and abraded it as thinly as possible with a high speed drill. The results were satisfactory. Sometimes, rupture of the dura mater did occur. In those cases, the dura mater needed repair.

Okada reported the en bloc method may induce postoperative spinal instability and preferred an open-door method [15]. However many authors reported en bloc method is safe and effective, with no postoperative spinal instability [16,26]. All patients in the present study underwent posterior thoracic laminectomy to remove the intruding ossified lesion. Efforts were made to preserve the lateral two thirds of the facet joints as much as possible to maintain the segmental stability. No postoperative instability was observed in our series. The key point is to preserve the lateral half of the facet. However, fluorosis makes the spine more rigid, decreases movement, and decreases the possibility of postoperative instability.

### Prognosis predictors

Several authors reported some factors influenced the surgical outcome which included preoperative neurological status, duration of preoperative symptoms, level and progression of ossification, and degree of thoracic kyphosis et al [27-30]. The result of our investigation confirmed that the preoperative JOA score is the most important predictor of the recovery rate. However, the duration of preoperative symptoms was not significantly correlated with the outcome. It might be because there were six patients who suffered acute onset of the symptom, just like acute spinal cord injury. The outcomes of these patients were not all good. To study this more, we divided all the patients into three groups according to preoperative symptom duration. Group one is acute onset, the duration shorter than three days. In group two, the symptom duration is between three days and five years. In group three, the symptom duration is longer than five years. ANOVA analysis of these three groups showed p = 0.0003. It showed that there was significant difference between the groups. Further t test showed that there was significant different between group one and group two (P = 0.0004). There was significant different between group two and group three (P = 0.003). However, there was no significant different between group one and group three (P = 0.197) (table 3). The result showed that the group with acute onset or too long duration had the worse surgical result.

The article "Thoracic myelopathy caused by ossification of ligamentum flavum of which fluorosis as an etiology factor" was retracted in 2007. Reasons: duplicate publication; a breach of policy by an author.

## Conclusion

Fluorosis can cause ossification of thoracic ligamentum flavum, as well as other ligaments. En bloc laminectomy decompression was an effective method. Preoperative JOA score was the most important predictor of surgical outcome. Patients with acute onset or too long duration had worse surgical outcome.
